The article "Antimalarial efficacy of Pongamia pinnata (L) Pierre against Plasmodium falciparum (3D7 strain) and Plasmodium berghei (ANKA)" was retracted in 2021. Reasons: duplicated images; original data or images not available; concerns about the data.

# Antimalarial efficacy of *Pongamia pinnata* (L) Pierre against *Plasmodium falciparum* (3D7 strain) and *Plasmodium berghei* (ANKA)

**DOI:** 10.1186/s12906-017-1958-y

**Published:** 2017-09-11

**Authors:** P.V.V. Satish, K. Sunita

**Affiliations:** Department of Zoology and Aquaculture, Acharya Nagarjuna University, Nagarjuna Nagar 522510, Guntur district, Andhra Pradesh India

**Keywords:** *Pongamia pinnata*, Antimalarial activity, Cytotoxicity evaluation, Phytochemical analysis, IC_50_, Selectivity index, Erythrocytic injury

## Abstract

**Background:**

The objective of the current study was to assess the in vitro antiplasmodial activities of leaf, bark, flower, and the root of *Pongamia pinnata* against chloroquine-sensitive *Plasmodium falciparum* (3D7 strain), cytotoxicity against Brine shrimp larvae and THP-1 cell line. For in vivo study, the plant extract which has shown potent in vitro antimalarial activity was tested against *Plasmodium berghei* (ANKA strain).

**Methods:**

The plant *Pongamia pinnata* was collected from the herbal garden of Acharya Nagarjuna University of Guntur district, Andhra Pradesh, India. Sequentially crude extracts of methanol (polar), chloroform (non-polar), hexane (non-polar), ethyl acetate (non-polar) and aqueous (polar) of dried leaves, bark, flowers and roots of *Pongamia pinnata* were prepared using Soxhlet apparatus. The extracts were screened for in vitro antimalarial activity against *P. falciparum* 3D7 strain. The cytotoxicity studies of crude extracts were conducted against Brine shrimp larvae and THP-1 cell line. Phytochemical analysis of the plant extracts was carried out by following the standard methods. The chemical injury to erythrocytes due to the plant extracts was checked. The in vivo study was conducted on *P. berghei* (ANKA) infected BALB/c albino mice by following 4-Day Suppressive, Repository, and Curative tests.

**Results:**

Out of all the tested extracts, the methanol extract of the bark of *Pongamia pinnata* had shown an IC_50_ value of 11.67 μg/mL with potent in vitro antimalarial activity and cytotoxicity evaluation revealed that this extract was not toxic against Brine shrimp and THP-1 cells. The injury to erythrocytes analysis had not shown any morphological alterations and damage to the erythrocytes after 48 h of incubation. Because methanolic bark extract of *Pongamia pinnata* has shown good antimalarial activity in vitro, it was also tested in vivo. So the extract had exhibited an excellent activity against *P. berghei* malaria parasite while decrement of parasite counts was moderately low and dose-dependent (*P* < 0.05) when compared to the control groups, which shown a daily increase of parasitemia, unlike the CQ-treated groups. The highest concentration of the extract (1000 mg/kg b.wt./day) had shown 83.90, 87.47 and 94.67% of chemo-suppression during Suppressive, Repository, and Curative tests respectively which is almost nearer to the standard drug Chloroquine (5 mg/kg b.wt./day). Thus, the study has revealed that the methanolic bark extract had shown promisingly high ((*P* < 0.05) and dose-dependent chemo-suppression. The phytochemical screening of the crude extracts had shown the presence of alkaloids, flavonoids, triterpenes, tannins, carbohydrates, phenols, coumarins, saponins, phlobatannins and steroids.

**Conclusions:**

The present study is useful to develop new antimalarial drugs in the scenario of the growing resistance to the existing antimalarials. Thus, additional research is needed to characterize the bioactive molecules of the extracts of *Pongamia pinnata* that are responsible for inhibition of malaria parasite.

## Background

The word malaria means ‘bad air’ which was originated from the Italian words ‘mal’ and ‘aria’ [1]. Malaria is an extremely dangerous parasitic disease infected by the protozoan parasites *Plasmodium falciparum*, *Plasmodium vivax*, *Plasmodium malariae* and *Plasmodium ovale.* Moreover, Plasmodium is transmitted to humans by the bite of infective Anopheles mosquito [2].

Malaria was widespread in the twentieth century in more than 100 countries throughout the tropical and subtropical zones including vast areas of Middle and South America, Hispaniola (Haiti and the Dominican Republic), Africa, Southeast Asia, Oceania and the Indian subcontinent. Drug resistance of *Plasmodium* to all traditional antimalarials and the insecticide resistance of mosquitoes and the finding of newly originated zoonotic parasite species has become problematical to prevent malaria [3].

The year 2015 was an extraordinary year for malaria control due to the three most hot news i.e., the Nobel Prize was given to Youyou Tu for the discovery of artemisinin, the development of first vaccine RTS,S against *P. falciparum* malaria and the fall of malaria infections worldwide particularly in sub-Saharan Africa. However, there are critical challenges that still deserve attention to boost malaria prevention and control due to the resistance of parasites to antimalarial drugs, and the RTS,S vaccines does not protect from *P. vivax* malaria and partially protect from *P. falciparum* malaria [4].

According to the WHO, malaria deaths declined in the year 2010 because of the extensive use of insecticide-coated mosquito nets and combination therapies of artemisinin derivatives [5]. In 2012, there were 207 million estimated cases of malaria in Africa and mortality was from 473,000 to 789,000 people and most of them were children under fifteen years [6].

The three most dangerous infectious diseases to human kind are AIDS, tuberculosis and malaria [7]. Despite every effort to eliminate the malaria infection, it remains one of the major infections facing by the people living in tropical and subtropical countries. The Indian subcontinent is known for *P. vivax* and *P. falciparum* infection, and most of the deaths reported were due to *P. falciparum* infection. Malaria has dramatically increased in India recently, after its near eradication in the early and mid-sixties [8].

Traditionally the plant extracts have always been considered as an important source in the medicine for treatment of malaria. Chloroquine, quinine, and artemisinin are the most effective antimalarial drugs derived from plants. The first successful antimalarial drug quinine was extracted from Cinchona tree; basing on this structure chloroquine and primaquine were derived. The current efficient antimalarial drug, Artemisinin was extracted from Chinese plant *Artemisia annua* in 1972 [9]. Artemisinin and its derivatives are used as first-line drugs to treat malaria according to World Health Organization. Regrettably, in 2009 artemisinin in resistance has been first reported in Thai-Cambodia border and accelerated the need for novel antimalarial drugs [10].

Now the World Health Organization has recommended artemisinin and its derivatives as single and in artemisinin combination with other drugs such as amodiaquine, lumefantrine, mefloquine, sulphadoxine- pyrimethamine (SP) as the first-line therapy for malaria worldwide [11]. As a result of this fact, the search for novel plant-derived antimalarial remedies began.

Thus the present investigation was focused to study the antimalarial activity of the plant *Pongamia pinnata*. *Pongamia pinnata* (L) Pierre commonly called as ‘Kanuga Tree,’ one of the most growing and popular plants of India. The ‘Pongamia’ name was originated from the Tamil, and ‘pinnata’ means ‘Pinnate leaves.’ This plant belongs to ‘Leguminosae’ family and its subfamily is ‘Papilionaceae.’ In Telugu (local language) this is known as ‘Ganuga’ or ‘Kanuga’. The plant is known as ‘Pungai,’ in Tamil, ‘Karanj’ in Hindi, ‘Karach’ in Bengali and ‘Pongamoil tree’ in English language.

*Pongamia pinnata* is a medium-sized ever green Indo-Malaysian species, commonly grown on alluvial and coastal habitats from India to Fiji, starting from sea level to 1200 m. Recently it is introduced in Florida, Australia, Malaysia, Hawaii, Seychelles, Philippines and Oceania as an exotic species. This plant stands as painted in crimson color in the months of March and April for about a week because of the buds developing with new leaves and then after the leaves grow mature, the tree acquires a beautiful bright lime-green color. *Pongamia pinnata* is predominantly cultivated in a large number of gardens and along with many roads in India and is becoming one of the most desirous trees of the city [12].

It has a number of phytochemical constituents belonging to a group of fixed oils and flavonoids. In folk medicine, sprouts and fruits of *Pongamia pinnata* are used as a remedy for tumors. Leaves are active against *Micrococcus,* due to the reason it is used for healing of cold, cough, dyspepsia, diarrhea, leprosy, flatulence and gonorrhea. The plant roots are mainly used for cleaning of teeth, teeth gums and ulcers. The bark is used as medicine for treatment of bleeding piles. Juices and oils of Pongamia are antibacterial and antiseptic. In the traditional medical practices like Unani and Ayurveda, the *Pongamia pinnata* plant and its parts are used for antiinflammatory, antiplasmodial, antilipidoxidative, antinonciceptive, antihyperglycaemic, antidiarrheal, antiulcer, antihyperammonic and antioxidantagent [13].

## Methods

### Collection of plant and its parts

Fresh samples of leaves, bark, flowers and roots of *Pongamia pinnata* were collected from Acharya Nagarjuna University’s Herbal Garden of Guntur district, Andhra Pradesh, India (Fig. 1). The confirmation of the plant species was done by Prof. S.M. Khasim, Department of Botany, Acharya Nagarjuna University, Guntur district, Andhra Pradesh, India. The voucher specimen of *Pongamia pinnata* was deposited in the Department of Botany, Acharya Nagarjuna University. All plant parts were washed immediately after collection with tap water and distilled water to remove the adhering organisms and dirt.

**Fig. 1:** Different plant parts of *Pongamia pinnata* used for the study

### Extract preparation

The methanol (polar), chloroform (non-polar), hexane (non-polar), ethyl acetate (non-polar) and aqueous or water (polar) crude extracts were prepared from shade-dried plant parts of leaves, bark, flowers and root in a Soxhlet apparatus (Borosil) at 50–60°C [14]. After complete extraction, the filtrates were concentrated separately by rotary vacuum evaporation (>45 °C) and then freeze dried (−20 °C) to obtain solid residue. The percent of extraction was calculated by using the following formula:

$$ Percentage\kern0.5em of\kern0.5em Extraction\kern0.5em =\kern0.5em \frac{Weight\kern0.5em of\kern0.5em the\kern0.5em extract\kern0.5em (g)}{Weight\kern0.5em of\kern0.5em the\kern0.5em plant\kern0.5em material\kern0.5em (g)}\times \kern0.5em 100 $$

The methanol, chloroform, hexane, ethyl acetate and aqueous extracts of leaf, bark, flower and root were screened for the presence of phytochemicals according to the method of Sofowora [15] and Kepam [16]. These extracts were then dissolved in dimethyl sulphoxide (DMSO) and were filtered through ‘millipore sterile filters’ (mesh 0.20 μm, Sartorious Stedim Biotech GmbH, Germany).

### Parasite cultivation

The *P. falciparum* strain was obtained from ongoing cultures in the departmental laboratory of the University. They were cultured according to the method of Trager and Jenson (1976) in candle jar desiccators. Then the *Plasmodium falciparum* culture was further cultivated in human O^Rh+^ red blood cells using RPMI 1640 medium (Sigma Laboratories Private Limited, Mumbai, India) supplemented with O^Rh+^ serum (10%), 5% sodium bicarbonate and 50 μg/mL of gentamycin sulfate. Hematocrits were adjusted at 2% and cultures of parasite were used when they exhibited 2% parasitemia [17].

### In vitro antimalarial screening (Simonsen et al., 2001)

The *P. falciparum* culture suspension of 3D7 (synchronized with 5% sorbitol to ring stage) was seeded (200 μL/well with 2% ring stages and 2% haematocrit) in 96-well tissue culture plates. The plant extracts (methanol, chloroform, hexane, ethyl acetate and aqueous extracts of leaf, bark, flower and root) of *Pongamia pinnata* were added to these wells in different concentrations (200, 100, 50, 25, and 12.5 μg/mL). Chloroquine treated parasites were kept as ‘control positive’ and DMSO treated parasites were kept as ‘control negative’ groups. The parasites were cultured for 30 h in candle jar desiccators. The cultures were incubated at 37°C for 48 h in an atmosphere of 2% O_2_, 5% CO_2_ and 93% N_2_. At 18 h before termination of the assay, [^3^H] Hypoxanthine (0.5 μCi/well) was added to each well. The effect of extracts in the cultures was evaluated by the measurement of [^3^H] Hypoxanthine incorporation into the parasite nucleic acids [18]. Each treatment has four replicates; at the end of the experiment, one set of the parasite infected red blood cells were collected from the wells, and blood smears were prepared. These smears were fixed with methanol and air dried. The smears were stained with Acridine Orange (AO) and Giemsa stain. Stained smears were observed under UV illumination microscope (Carl Zeiss) for confirmation of [^3^H] Hypoxanthine assay. The experiment was terminated and the cultures were frozen and stored at −20°C. The parasites were harvested on glass filter papers using NUNC Cell Harvester and CPM (count per minute) was recorded in gamma scintillation counter. Control readings were considered to be as 100% parasite growth and the parasite inhibition was calculated for plant extract treated samples. The parasite inhibition was calculated as follows (19):

$$ \%\kern0.5em Inhibition=\frac{Average\kern0.5em CPM\kern0.5em of\kern0.5em Control\kern0.5em -\kern0.5em Average\kern0.5em CPM\kern0.5em of\kern0.5em plant\kern0.5em extract}{Average\kern0.5em CPM\kern0.5em of\kern0.5em Control}\times \kern0.5em 100 $$

The IC_50_ values were determined by plotting concentration of extract on X-axis and percentage of inhibition on Y-axis with dose-response curves using Minitab 11.12.32. Bit software.

The in vitro antiplasmodial activity of the extracts was categorized into four groups based on IC_50_ value i.e., <5 μg/mL - very active, 5–50 μg/mL - active, 50–100 μg/mL - weakly active, >100 μg/mL - inactive [19].

### Brine shrimp lethality assay (BSLA) (in vivo assay)

In the present study, the brine shrimp larvae were collected from hatched eggs of *Artemia salina* cultured in artificial sea water (20 g NaCl and 18 g table salt in 1 l of distilled water) for 24 h at room temperature (25–30°C).The crude extracts (methanol, chloroform, hexane, ethyl acetate and aqueous extracts of leaf, bark, flower and root) of *Pongamia pinnata* were dissolved in DMSO in different concentrations of 100, 200, 400, 600, 800, 1000, 1200, 1400, 1600 and 1800 μg/mL were added to each test tube containing 10 live nauplii in 10 mL of artificial sea water. The solvent (DMSO) concentration was not more than 5% and had no adverse effects on the larvae. The same procedure was followed for the standard drug chloramphenicol (control positive) and the final volume for each test tube was made up to 10 ml with artificial sea water with ten live nauplii in each test tube. The ‘control negative’ test tube with DMSO contained 10 live nauplii in 10 mL of artificial sea water. After 24 h, the test tubes were observed and the number of survived nauplii in each test tube was counted and the results were noted. The percentage of dead nauplii in the test and the standard group was established by comparing with that of the control group. The percentage of mortality was plotted against log concentrations, and the lethal concentrations (LC_50_) was deliberated by Finney’s probit analysis [20]. The general toxicity activity was considered weak when the LC_50_ ranged from 500 μg/mL to 1000 μg/mL, moderate when the LC_50_ ranged from 100 μg/mL to 500 μg/mL and strong when the LC_50_is ≤ 100 μg/mL [21]. In vivo selectivity index (SI) was determined for each extract as follows:

$$ SI\kern0.5em =\kern0.5em \frac{LC50\kern0.5em of\kern0.5em Brine\kern0.5em shrimp}{LC50\kern0.5em of\kern0.5em P.\kern0.5em falciparum} $$

### Cytotoxicity of extracts to THP-1 monocyte cells

Cytotoxicity studies of the crude extracts (methanol, chloroform, hexane, ethyl acetate and aqueous extracts of leaf, bark, flower and root) of *Pongamia pinnata* were conducted by functional assay using THP-1 cells [22]. 10% fetal bovine serum, 0.21% sodium bicarbonate (Sigma), and 100 μg/mL penicillin and 50 μg/mL gentamicin (complete medium) containing RPMI-1640 (Roswell Park Memorial Institute 1640) medium was used for the culture of cells. Briefly, cells (0.2 × 10^6^ cells/200 μL/well) were seeded into 96-well culture plates in complete medium. The plant extracts (200, 100, 50, 25 and 12.5 μg/mL) were added after 24 h of seeding and incubated for 48 h in a humidified atmosphere at 37 °C and 5% CO_2_. DMSO and ellipticine were kept as control negative and control positive respectively. After termination of the experiments 10 μL of MTT stock solution (5 μg/mL in 1× PBS) was added to each well, gently mixed and incubated for another four hours. The plates were centrifuged at 1500 rpm for 5 min; the supernatants were discarded, subsequently added 100 μL of DMSO (stopping agent) in each well. After formation of formazan, it was read on a microtiter plate reader (Versa max tunable multi well plate reader) at 570 nm, and the percentage of cell viability was calculated using the following formula [23].

$$ \%\kern0.5em Cell\kern0.5em Viability\kern0.5em =\kern0.5em \frac{Mean\kern0.5em absorbance\kern0.5em in\kern0.5em test\kern0.5em wells}{Mean\kern0.5em absorbance\kern0.5em in\kern0.5em control\kern0.5em wells}\kern0.5em \times \kern0.5em 100 $$

The SI of in vitro toxicity was calculated for each extract using the following formula:

$$ SI\kern0.5em =\kern0.5em \frac{IC50\kern0.5em THP-1\kern0.5em cells}{IC50\kern0.5em of\kern0.5em P.\kern0.5em falciparum} $$

The IC_50_ values were determined by plotting the concentration of extract on X-axis and percentage of cell viability on Y-axis with dose-response curves using Minitab 11.12.32. Bit software.

### Chemical injury to erythrocytes

To assess the chemical injury to erythrocytes due to the plant extracts (methanol, chloroform, hexane, ethyl acetate and aqueous extracts of leaf, bark, flower and root) of *Pongamia pinnata*; 200 μL of erythrocytes were incubated with 200 μg/mL of the extract, a dose equal to that of the highest dose used in the antiplasmodial assay. The experiments were conducted under the same conditions as that of the antiplasmodial assay. After 48 h of incubation, the assay was terminated and thin blood smears were prepared and fixed with methanol and air dried. These smears were stained with Giemsa stain and observed for morphological variations of erythrocytes if any, under a light microscope. These morphological findings were compared with the normal erythrocytes of the control group [24].

### Extracts dilutions

The methanol, chloroform, hexane, ethyl acetate and aqueous extracts of leaves, bark, flowers and roots of *Pongamia pinnata* were first dissolved in DMSO to prepare a stock concentration of 50 mg/mL. Then the stock solution was diluted in RPMI 1640 medium to make 10 mg/mL of working concentration for in vitro (*P. falciparum* and THP-1 cells) studies. From the above working solution, different concentrations of crude extracts (methanol, chloroform, hexane, ethyl acetate and aqueous extracts of leaf, bark, flower and root) such as 12.5, 25, 50, 100 and 200 μg/mL were prepared by serial dilution [25] for antimalarial screening against CQ-sensitive *P. falciparum* 3D7 strain and to test cytotoxicity against THP-1 cell line.

Moreover, a working solution of 50 mg/mL was prepared for in vivo (brine shrimp and mice) studies. The concentrations from 100 to 1600 μg/mL were prepared by serial dilution for toxicity against brine shrimp. The plant extract concentrations from 200 to 1000 mg/kg were prepared with PBS (phosphate buffered saline) for in vivo antimalarial activity against *P. berghei* in BALB/c mice.

### In vivo study of Methanolic bark extract

Healthy BALB/c female mice of age 6–8 weeks (25–30 g) were used for the present investigation. The mice were fed on standard pellet diet and water was given ad libitum. They were kept in clean, dry polypropylene cages and maintained in a well-ventilated animal house with 12 h light/12 h dark cycle. Animal experiments were conducted according to the guidelines of Institutional Animal Ethics Committee of Hindu College of Pharmacy, Guntur (IAEC Ref. No. HCOP/IAEC/PR-21/2014), Andhra Pradesh, India.

The chloroquine sensitive *Plasmodium berghei* ANKA strain was maintained in vivo in BALB/c mice in our laboratory by weekly inoculation of 1 × 10^7^ infected red blood cells in naïve mice. Then the parasitemia was counted with a hemocytometer and adjusted the parasites 0.5 × 10^6^ in PBS sterile solution. Each animal was injected intraperitoneally (IP) with 200 μL (0.2 mL) with 0.5×10^6^ parasites inoculated on the first day i.e., day-0 [26].

For evaluating the methanol bark crude extract, infected mice were randomly divided into seven groups of 3 mice per group. Group I to Group V were treated with the methanol bark extract (most effective among all the other extracts) of *Pongamia pinnata* at doses of 200 mg/kg, 400 mg/kg, 600 mg/kg, 800 mg/kg and 1000 mg/kg respectively. The remaining two groups were maintained as control negative and control positive; and administered PBS and chloroquine with 5 mg/kg body weight/day respectively.

### The 4-day suppressive test

This test was used to evaluate the schizonticidal activity of the methanolic extract of the bark of *Pongamia pinnata* against *P. berghei* infected mice according to the method described by Peter et al. [27]. These infected mice were randomly divided into the respective groups as described above. Then the treatment was started three hours after mice had been inoculated with the parasites on day-0 and then continued daily for four days from day-0 to day-3. After completion of treatment, thin blood film was prepared from the tail of each animal on day-4 to determine parasitemia and percentage of inhibition. Additionally, each mouse was observed daily for determination of survival time.

### Evaluation of the repository activity

Evaluation of repository activity was conducted according to the method described by Peter et al. [27]. Initially, five groups of mice (3 mice in each group) were administered intraperitoneally (IP) with the methanolic extract of the bark of *Pongamia pinnata*, chloroquine (control positive) and PBS (control negative) for four consecutive days (D0-D3) respectively as described above. On the fifth day (D4), the mice were inoculated with *Plasmodium berghei* infected red blood cells. Seventy-two hours later, the parasitemia level was evaluated by observing Giemsa-stained blood smears. Also, the mice were observed during the study period for determination of survival time.

### Rane’s Test or curative test

To evaluate the curative potential of the methanolic crude extract of bark of *Pongamia pinnata*, the most active fraction in Peter’s test was evaluated according to the method described by Ryley and Peters [28]. On day-0, a standard inoculums of 0.5×10^6^ infected erythrocytes was inoculated into each mouse intraperitoneally (IP). After seventy-two hours, mice were randomly divided into their respective groups and administrated the extract once daily for five days. Giemsa-stained thin blood film was prepared from the tail of each mouse daily for five days to monitor parasitemia level. Mean survival time for each group was determined arithmetically by calculating the average survival time (days) of mice starting from the date of infection over a period of 30 days (D0-D29).

### Parasitemia measurement

Thin smears of blood were made from the tail of each mouse at the end of each test. The smears were prepared on glass slides (76 × 26 mm), fixed with absolute methanol for 15 min and stained with 10% Giemsa stain at pH 7.2 for 15 min. And were also stained with Acridine Orange. The stained slides were then washed gently using distilled water and air dried at room temperature. Two stained slides for each mouse were examined under a Trinocular microscope (CHi20) and UV illumination microscope (Carl Zeiss) under 1000× magnification. Ten fields on each slide were observed to calculate the percent of parasitemia [29].

$$ Parasitemia\kern0.5em \left(\%\right)\kern0.5em =\frac{No.\kern0.5em parasitized\kern0.5em RBC}{Total\kern0.5em No.\kern0.5em of\kern0.5em RBC}\times \kern0.5em 100 $$

Also the percentage of parasitemia suppression due to the effect extracts was calculated using the following formula.

$$ Suppression\kern0.5em \left(\%\right)\kern0.5em =\kern0.5em \frac{Mean\kern0.5em parasitemia\kern0.5em of\kern0.5em control\kern0.5em negative\kern0.5em group}{Mean\kern0.5em parasitemia\kern0.5em of\kern0.5em treated\kern0.5em group}\times \kern0.5em 100 $$

### Monitoring of body weight

For Peter’s test, the body weight of each mouse was measured before infection (day 0) and on day 4 using a sensitive digital weighing balance. For Rane’s test, body weight was measured before infection and from day 3–7 after infection. For repository test, body weight was measured before dosing periods and on dosing periods.

### Packed cell volume measurement

Packed cell volume (PCV) was measured to predict the effectiveness of the test extract in preventing hemolysis resulting from increasing parasitemia associated with malaria. Heparinized capillary tubes were used for collection of blood from the tail of each mouse. The capillary tubes were filled with blood up to ¾^th^ of their volume and sealed at the dry end with sealing clay. The tubes were then placed in a micro-haematocrit centrifuge with the sealed end outwards and centrifuged for 5 min at 11,000 rpm. The tubes were then taken out of the centrifuge and PCV was determined using a standard Micro-Hematocrit Reader. The PCV is a measure of the proportion of RBCs to plasma and measured before inoculating the parasite and after treatment using the following formula [30]:

$$ PCV\kern0.5em \left(\%\right)\kern0.5em =\kern0.5em \frac{Volume\kern0.5em of\kern0.5em erythrocytes\kern0.5em in\kern0.5em given\kern0.5em volume\kern0.5em of\kern0.5em blood}{Total\kern0.5em blood\kern0.5em volume}\times \kern0.5em 100 $$

### Statistical analysis

The mean and standard deviations of the treated and control groups were calculated at 95% confidence intervals for inhibition, mortality, parasitemia, body weight and PCV. The results were analyzed statistically by two-tailed student’s t-test to identify the differences between the treated group and control group with Minitab 11.12.32. Bit software. The data was considered significant at *P* < 0.05.

## Results

### Yield of crude extracts from *Pongamia pinnata* and it’s phytochemicals

The weight of leaves, bark, flowers and roots extracts of *Pongamia pinnata* in methanol, chloroform, hexane, ethyl acetate and aqueous respectively were shown in Table 1. The percent yield of extracts varied from 1.48% to 15.32%. It was revealed that, chloroform extract of flowers (15.32%) shown highest percent yield followed by hexane extract of leaves (14.90%). The phytochemical screening has revealed the presence of various phytochemical compounds in the methanol, chloroform, hexane, ethyl acetate and aqueous extracts of leaves, bark, flowers and roots of *Pongamia pinnata.* But flavonoids are the common phytochemicals found in the extracts excepting in the root extracts (Table 2).

**Table 1:** Weight and percentage yield of different crude extracts of *Pongamia pinnata*

Plant part	Extract	Wight of plant part (g)	Wight of extract yield (g)	Yield (%)
Leaf	ME	50	3.24	6.48
	CH	50	4.54	9.08
	HE	50	7.45	14.90
	EA	50	0.74	1.48
	AQ	50	2.27	4.54
Bark	ME	50	2.23	4.46
	CH	50	4.56	9.12
	HE	50	7.11	14.22
	EA	50	1.27	2.54
	AQ	50	3.51	7.02
Flower	ME	50	4.51	9.02
	CH	50	7.66	15.32
	HE	50	6.08	12.16
	EA	50	1.33	2.66
	AQ	50	3.54	7.08
Root	ME	50	2.23	4.46
	CH	50	2.98	5.96
	HE	50	6.21	12.42
	EA	50	1.92	3.84
	AQ	50	2.22	4.44

*ME* Methanol, *CH* Chloroform, *HE* Hexane, *EA* Ethyl acetate, *AQ* Aqueous

**Table 2:** Phytochemical constituents of *Pongamia pinnata* in different extracts of leaf, bark, flower and root

Tested compounds	Leaf					Bark					Flower					Root				
	ME	CH	HE	EA	AQ	ME	CH	HE	EA	AQ	ME	CH	HE	EA	AQ	ME	CH	HE	EA	AQ
Alkaloids	–	–	–	+	–	–	–	–	+	–	–	–	–	+	–	–	–	–	–	–
Coumarins	+	–	–	–	–	+	–	–	–	–	–	–	–	+	–	+	–	–	–	–
Carbohydrates	–	–	–	–	+	–	–	–	–	+	–	–	–	–	+	–	–	–	–	–
Phenols	+	–	–	+	–	–	–	–	+	–	+	–	–	+	–	+	–	+	–	–
Saponins	–	+	–	+	–	–	+	–	–	–	+	–	–	+	–	+	–	–	–	–
Tannins	+	–	–	+	–	+	–	–	+	–	+	–	–	–	+	+	–	–	–	–
Flavonoids	+	+	+	+	+	+	–	+	–	+	–	–	–	+	+	–	–	–	–	–
Terpenoids	+	–	–	–	–	+	+	–	–	–	+	–	–	+	–	+	–	–	–	–
Phlobatannins	–	–	–	+	–	–	–	–	–	–	–	–	–	+	–	–	–	+	+	–
Steroids	–	+	+	–	–	–	+	+	–	–	–	+	+	–	–	–	+	+	–	–

+ Present, − Absent, ME- Methanol, CH- Chloroform, HE- Hexane, EA- Ethyl acetate, AQ- Aqueous

### In vitro antimalarial activity

The present experimentation evaluated the antimalarial activity of the crude extracts of methanol, hexane, chloroform, ethyl acetate and aqueous from leaves, bark, flowers and roots of *Pongamia pinnata.* The IC_50_ values of the plant extracts tested against *Plasmodium falciparum* are shown in Table 3.

**Table 3:** Antiplasmodial activity against *P. falciparum* 3D7 strain of different crude extracts from *Pongamia pinnata*

Plant Part	Extract	Percentage of inhibition (M ± SD, *P* value)					IC_50_ (μg/mL) 95% *CI* (LCL-UCL)
		12.5 μg/mL	25 μg/mL	50 μg/mL	100 μg/mL	200 μg/mL	
Leaf	ME	21.08 ± 2.21 0.0019	49.78 ± 0.88 0.0001	68.75 ± 3.20 0.0004	86.85 ± 1.08 0.0000	95.01 ± 3.97 0.0003	24.00 ± 1.00 (21.51–26.48)
	CH	0.00 ± 0.00 NS	0.00 ± 0.00 NS	0.00 ± 0.00 NS	2.59 ± 1.46 0.12^NS^	2.75 ± 0.83 0.78 ^NS^	ND
	HE	0.00 ± 0.00 NS	0.00 ± 0.00 NS	1.22 ± 0.115 0.0023	2.49 ± 0.58 0.037	3.09 ± 0.17 0.76 ^NS^	ND
	EA	13.18 ± 2.56 0.0063	26.84 ± 2.22 0.0012	38.33 ± 5.92 0.0040	67.19 ± 3.37 0.0004	72.28 ± 2.22 0.0002	70.33 ± 3.79 (60.93–79.74)
	AQ	8.23 ± 0.96 0.0024	14.38 ± 4.31 0.015	27.08 ± 1.22 0.0003	54.07 ± 4.46 0.0012	78.07 ± 4.08 0.0005	92.00 ± 7.00 (74.61–109.39)
Bark	ME	51.18 ± 3.57 0.0008	88.07 ± 0.80 0.0000	97.21 ± 1.00 0.0000	98.40 ± 0.32 0.0000	100 ± 0.12 0.0000	11.67 ± 1.53 (7.87–15.46)
	CH	0.00 ± 0.00 NS	5.54 ± 0.62 0.0022	18.02 ± 2.38 0.0029	27.31 ± 2.04 0.0010	41.67 ± 1.34 0.0002	>200
	HE	0.00 ± 0.00 NS	6.50 ± 1.63 0.0011	17.25 ± 0.90 0.0005	34.52 ± 3.73 0.0021	54.12 ± 3.50 0.0008	178.41 ± 14.74 (141.71–214.96)
	EA	11.19 ± 2.65 0.0093	25.84 ± 3.31 0.0027	52.49 ± 2.12 0.0003	78.41 ± 3.49 0.0003	85.20 ± 2.60 0.0002	46.57 ± 1.53 (42.87–50.46)
	AQ	15.51 ± 1.95 0.0027	34.34 ± 3.56 0.0018	65.42 ± 0.73 0.0000	90.44 ± 1.18 0.0000	98.37 ± 0.26 0.0000	37.18 ± 1.53 (33.54–41.13)
Flower	ME	14.22 ± 3.47 0.0098	39.70 ± 1.93 0.0004	67.21 ± 1.02 0.0000	93.42 ± 2.82 0.0002	97.58 ± 0.88 0.0000	32.00 ± 2.00 (27.03–36.97)
	CH	0.00 ± 0.00 NS	5.55 ± 0.49 0.0014	16.49 ± 1.89 0.0022	34.37 ± 3.65 0.0020	62.12 ± 0.25 0.0000	156.10 ± 3.61 (147.04–164.96)
	HE	3.11 ± 0.10 0.0003	10.01 ± 1.21 0.0025	28.58 ± 2.05 0.0009	35.52 ± 2.72 0.0011	43.50 ± 2.96 0.0009	>200
	EA	7.33 ± 1.65 0.0086	19.57 ± 0.77 0.0003	46.62 ± 1.88 0.0003	67.34 ± 0.81 0.0000	81.72 ± 1.23 0.0000	58.00 ± 4.58 (46.62–69.39)
	AQ	10.51 ± 0.90 0.0013	38.01 ± 0.88 0.0001	55.31 ± 4.88 0.0013	81.29 ± 1.05 0.0000	94.02 ± 1.42 0.0000	42.43 ± 3.21 (34.35–50.32)
Root	ME	25.17 ± 2.23 0.0013	48.28 ± 0.92 0.0001	62.82 ± 2.31 0.0002	78.87 ± 5.80 0.0009	92.15 ± 3.68 0.0003	25.67 ± 2.08 (20.50–30.84)
	CH	2.44 ± 0.68 0.014	8.80 ± 2.00 0.0087	20.57 ± 0.87 0.0003	44.27 ± 3.56 0.0011	68.63 ± 1.16 0.0001	123.77 ± 10.26 (98.17–149.16)
	HE	0.00 ± 0.00 NS	0.00 ± 0.00 NS	0.00 ± 0.00 NS	1.90 ± 0.54 0.092 ^NS^	2.65 ± 0.67 0.86 ^NS^	ND
	EA	0.00 ± 0.00 NS	0.00 ± 0.00 NS	1.81 ± 0.55 0.017	2.14 ± 0.17 0.0074	2.53 ± 0.54 0.93 ^NS^	ND
	AQ	1.30 ± 0.23 0.0072	7.47 ± 1.11 0.0038	23.31 ± 1.11 0.0004	58.04 ± 0.34 0.0000	69.38 ± 1.76 0.0001	88.00 ± 1.73 (83.70–92.90)
DMSO (Negative control)	–	0.55 ± 0.01	1.32 ± 0.31	2.35 ± 0.00	4.16 ± 0.14	4.00 ± 0.64	–
CQ (Positive control)	–	–	–	–	–	–	3.68 ± 0.555

Values are represented as mean of 3 replicates ± standard deviation at 95% confidence intervals with lower and upper limits and *P* - value is significant at <0.05 and <0.001, NS- not significant, ME- methanol, CH- chloroform, HE- hexane, EA- ethyl acetate, AQ- aqueous, DMSO- Dimethyl sulphoxide, CQ- chloroquine

The IC_50_ value of the methanol, chloroform, hexane, ethyl acetate and aqueous extracts of leaves, bark, flowers and roots of *Pongamia pinnata* showed a range (IC_50_ = 11.67 μg/mL to 178.41 μg/mL) of inhibitory concentrations against CQ-sensitive *P. falciparum* strain.

The methanolic extract of leaves (24.00 μg/mL), bark (11.67 μg/mL), flowers (32 .00 μg/mL) and roots (25.77 μg/mL); aqueous extract of bark (37.18 μg/mL), flowers (42.42 μg/mL) and ethyl acetate extract of bark (46.57 μg/mL) showed IC_50_ values <50 μg/mL which were significant at *P* < 0.05 indicating good antimalarial activity. Among these extracts methanol extract of bark showed very minimal IC_50_ value (11.67 μg/mL) showing better antimalarial activity than the other extracts [19].

The ethyl acetate extracts of leaves (70.33 μg/mL) and flowers (58.00 μg/mL); the aqueous extracts of leaves (92.00 μg/mL) and roots (88.00 μg/mL) showed IC_50_ values between 50 and 100 μg/mL indicating weak antimalarial activity.

The chloroform extract of bark and hexane extract of flower showed IC_50_ values greater than 200 μg/mL indicating inactivity against malaria parasite. And the IC_50_ values of chloroform and hexane extracts of leaves and roots were not determinate due to their unclear inhibition [19].

Out of the 20 extracts tested; seven extracts have shown active (IC_50_ = 11.67 to 46.57 μg/mL) antimalarial activity, four extracts have shown weak (IC_50_ = 58.00 to 92.00 μg/mL) antimalarial activity, while nine extracts have no antimalarial activity (IC_50_ = >100 μg/mL). Thus methanolic extract of bark has shown very minimal IC_50_ value (11.67 μg/mL) with excellent antimalarial activity when compared to the activity of other tested extracts.

The microscopic observation of inhibition of *Plasmodium falciparum* by treatment with methanolic extracts (200 μg/mL) is shown in Figs. 2 and 3. The CPM values after the treatment of all the extracts at the highest concentration of 200 μg/mL are represented in Fig. 4.

**Fig. 2:** Microscopic observations after treatment with methanolic extracts of *Pongamia pinnata* against *P. falciparum* 3D7 strain at the highest concentration (200 μg/mL) with Acridine Orange stain at 1000× magnification (R- ring stage, T- trophozoite, S- schizont)

**Fig. 3:** Microscopic observations after treatment with methanolic extracts of *Pongamia pinnata* against *P. falciparum* 3D7 strain at the highest concentration (200 μg/mL) with Giemsa stain at 1000× magnification (R- ring stage, T- trophozoite, S- schizont)

**Fig. 4:** Counts per minute (CPM) of untreated (control) and treated groups against *P. falciparum* 3D7 strain

### Cytotoxicity evaluation against brine shrimp

During cytotoxicity evaluation the methanol, chloroform, hexane, ethyl acetate and aqueous extracts of leaves, bark, flowers and roots showed LC_50_ values between 480.00 μg/mL to 1475.00 μg/mL. In general, the extracts are considered as nontoxic when the LC_50_ > 1000 μg/mL, weak when the LC_50_ is between 500 μg/mL to 1000 μg/mL, moderate when LC_50_ is between 100 μg/mL to 500 μg/mL and strong when the LC_50_ is <100 μg/mL. Based on the above classification, out of the 20 extracts tested, 11 extracts were nontoxic (LC_50_ > 1000 μg/mL), 6 extracts displayed weak (LC_50_ 500–1000 μg/mL) toxicity, 3 extracts exhibited moderate toxicity (LC_50_ 100–500 μg/mL) and none of the extracts showed LC_50_ < 100 μg/mL as indicated in Table 4. The SI values were calculated and most of the extracts showed SI value >10 indicating that the extracts are safer for further studies.

**Table 4:** Cytotoxicity against brine shrimp larva of different crude extracts from *Pongamia pinnata*

Plant Part	Extract	Percentage of mortality (M ± SD, *P* - value)								LC_50_ (μg/mL) 95%*CI* (LCL-UCL)		SI
		100 μg/mL	200 μg/mL	400 μg/mL	600 μg/mL	800 μg/mL	1000 μg/mL	1200 μg/mL	1400 μg/mL	1600 μg/mL		
Leaf	ME	0.00 ± 0.00 NS	4.74 ± 1.45 0.017	10.52 ± 2.93 0.013	18.15 ± 2.63 0.0036	30.53 ± 0.62 0.0001	38.87 ±1.65 0.0003	45.33 ±3.51 0.0013	69.45 ±5.03 0.0012	87.61 ± 1.58 0.0001	1245.00 ±35.00 (1158.10–1331.90)	51.87
	CH	7.37 ± 0.50 0.0009	13.38 ± 0.94 0.0009	24.02 ± 1.13 0.0004	38.37 ± 4.17 0.0020	56.25 ± 0.97 0.0001	82.62 ±2.18 0.0001	100.00 ±0.00 0.0000	100.00 ±0.00 0.0000	100.00 ±0.00 0.0000	730.00 ±22.9 1030.80–1182.60)	ND
	HE	0.00 ± 0.00 NS	4.15 ±0.37 0.0020	10.69 ±1.70 0.0011	18.33 ±1.55 0.0013	38.33 ±1.66 0.0003	41.22 ±0.91 0.0001	56.61 ±3.15 0.0006	74.36 ±4.48 0.0008	97.57 ±2.12 0.0001	1106.70 ±30.60 (1030.80–1182.60)	ND
	EA	10.70 ±1.57 0.0039	18.48 ±0.96 0.0005	37.62 ±4.10 0.0020	61.82 ±1.39 0.0001	86.04 ±3.04 0.0002	100.00 ±0.00 0.0000	100.00 ±0.00 0.0000	100.00 ±0.00 0.0000	100.00 ±0.00 0.0000	495.00 ±22.90 (438.10–551.90)	7.03
	AQ	13.06 ±1.47 0.0022	25.32 ±2.66 0.0019	46.50 ±1.28 0.0001	61.96 ±1.99 0.0002	90.87 ±1.72 0.0001	100.00 ±0.00 0.0000	100.00 ±0.00 0.0000	100.00 ±0.00 0.0000	100.00 ±0.00 0.0000	438.00 ±10.58 (411.71–464.29)	4.76
Bark	ME	0.00 ±0.00 NS	0.00 ±0.00 NS	2.31 ±0.31 0.0013	7.74 ±2.26 0.015	13.13 ±2.23 0.0050	21.22 ±2.02 0.0018	38.79 ±1.73 0.0005	55.51 ±5.04 0.0021	85.00 ±0.37 0.0000	1328.30 ±32.50 (1247.50–1409.10)	113.82
	CH	0.00 ±0.00 NS	3.30 ±1.20 0.026	9.82 ±2.26 0.0093	15.03 ±1.60 0.0020	26.78 ±2.59 0.0017	48.37 ±0.80 0.0001	69.53 ±3.60 0.0005	88.29 ±0.52 0.0000	100.00 ±0.00 0.0000	1011.67 ±2.89 (1004.50–1018.84)	>5.05
	HE	5.23 ±0.38 0.0012	9.49 ±1.06 0.0023	16.62 ±3.80 0.0089	38.08 ±0.94 0.0001	54.55 ±3.66 0.0008	72.60 ±2.24 0.0002	91.70 ±3.79 0.0003	98.18 ±1.21 0.0001	100.00 ±0.00 0.0000	738.30 ±23.60 (679.60–797.00)	4.14
	EA	0.00 ±0.00 NS	4.23 ±0.68 0.0054	10.67 ±3.19 0.015	18.08 ±0.92 0.0005	42.01 ±3.09 0.0010	74.07 ±0.82 0.0000	98.15 ±2.48 0.0001	100.00 ±0.00 0.0000	100.00 ±0.00 0.0000	841.37 ±10.41 (815.81–867.52)	18.02
	AQ	0.00 ±0.00 NS	1.30 ±0.24 0.0056	4.53 ±1.51 0.020	10.49 ±0.70 0.0008	22.53 ±4.07 0.0054	49.02 ±1.63 0.0003	80.37 ±2.85 0.0002	100.00 ±0.00 0.0000	100.00 ±0.00 0.0000	1006.00 ±14.93 (968.90–1043.10)	26.94
Flower	ME	0.00 ±0.00 NS	0.00 ±0.00 NS	0.00 ±0.00 NS	0.00 ±0.00 NS	3.37 ±0.17 0.017	11.03 ±1.84 0.0069	21.83 ±1.51 0.0016	38.59 ±2.95 0.0019	66.10 ±3.63 0.0007	1475.00 ±21.80 (1420.90–1529.01)	46.09
	CH	0.00 ±0.00 NS	0.00 ±0.00 NS	3.31 ±0.82 0.013	7.71 ±1.21 0.0045	15.25 ±2.39 0.0048	29.41 ±0.74 0.0001	47.34 ±1.75 0.0003	68.61 ±3.95 0.0008	84.66 ±3.83 0.0005	1218.33 ±10.41 (1192.48–1244.19)	7.80
	HE	0.00 ±0.00 NS	1.56 ±0.50 0.029	4.07 ±1.34 0.020	12.46 ±2.80 0.0087	31.78 ±2.12 0.0008	58.65 ±2.03 0.0002	75.79 ±1.98 0.0001	91.41 ±1.17 0.0000	100.00 ±0.00 0.0000	1132.67 ±15.53 (1094.08–1171.26)	>5.66
	EA	9.11 ±1.95 0.0081	17.54 ±4.05 0.0090	33.32 ±2.73 0.0011	71.34 ±2.87 0.0003	89.30 ±0.29 0.0000	99.34 ±0.28 0.0000	100.00 ±0.00 0.0000	100.00 ±0.00 0.0000	100.00 ±0.00 0.0000	480.00 ±5.00 (467.58–492.42)	8.27
	AQ	6.21 ±0.89 0.0039	10.89 ±2.16 0.0069	21.51 ±1.26 0.0006	38.76 ±3.90 0.0017	59.91 ±3.75 0.0007	78.20 ±0.96 0.0000	99.30 ±0.34 0.0000	100.00 ±0.00 0.0000	100.00 ±0.00 0.0000	703.30 ±28.40 (632.70–774.00)	16.61
Root	ME	0.00 ±0.00 NS	0.00 ±0.00 NS	0.00 ±0.00 NS	2.41 ±0.66 0.017	6.77 ±1.88 0.018	14.37 ±2.11 0.0048	38.32 ±1.19 0.0003	69.20 ±1.03 0.0000	90.89 ±1.72 0.0001	1274.00 ±5.29 (1260.86–1287.14)	49.62
	CH	0.00 ±0.00 NS	0.00 ±0.00 NS	0.00 ±0.00 NS	3.83 ±0.44 0.0031	10.47 ±0.45 0.0004	18.51 ±0.49 0.0011	32.79 ±2.33 0.0013	58.88 ±3.11 0.0007	89.30 ±2.60 0.0002	1335.00 ±21.80 (1280.90–1389.10)	10.79
	HE	0.00 ±0.00 NS	2.48 ±1.13 0.042	8.41 ±0.96 0.0024	18.74 ±3.16 0.0049	39.78 ±2.49 0.0007	80.13 ±1.81 0.0001	99.15 ±0.17 0.0000	100.00 ±0.00 0.0000	100.00 ±0.00 0.0000	850.17 ±5.21 (828.26–873.07)	ND
	EA	3.45 ±0.59 0.0066	9.09 ±3.15 0.020	19.27 ±0.49 0.0001	40.65 ±2.78 0.0008	78.34 ±0.82 0.0000	96.68 ±1.87 0.0001	100.00 ±0.00 0.0000	100.00 ±0.00 0.0000	100.00 ±0.00 0.0000	646.72 ±15.28 (608.12–684.61)	ND
	AQ	0.00 ±0.00 NS	0.00 ±0.00 NS	2.32 ±0.13 0.0003	6.62 ±2.00 0.016	13.44 ±3.02 0.0098	42.58 ±2.04 0.0004	73.39 ±3.36 0.0004	98.04 ±0.95 0.0000	100.00 ±0.00 0.0000	1047.61 ±12.50 (1016.61–1078.73)	11.90
DMSO (−ve control)	–	0.80 ± 0.03	1.00 ±0.21	1.12 ±0.00	1.47 ±0.52	1.50 ±0.00	2.31 ±0.17	4.33 ±0.38	5.45 ±0.59	7.87 ±1.21	–	–
Chloram-phenicol (+ve control)	–	–	–	–	–	–	–	–	–	–	19.45 ±1.23	

Values are represented as mean of 3 replicates ± standard deviations at 95% confidence interval with upper and lower limits and *P* - value is significant at <0.05 and <0.001, NS– not significant; ME- methanol, CH- chloroform, HE- hexane, EA- ethyl acetate, AQ- aqueous; SI- selective index (SI = LC_50_ Brine shrimp larva /IC_50_ *P. f* 3D7 strain), DMSO- Dimethyl sulphoxide, CQ- chloroquine

### Cytotoxicity evaluation against THP-1 cells

The cytotoxicity studies of twenty different extracts against THP-1 cell line shown IC_50_ values >200 μg/mL. An extract was considered as non-toxic if the IC_50_ was >20 μg/mL. Based on the above, the plant extracts were non-toxic and can be used for further investigations. The SI values were also calculated and listed in Table 5.

**Table 5:** Cytotoxocity against THP-1 cell line of different crude extracts from *Pongamia pinnata*

Plant Part	Extract	Percentage of Inhibition (M ± SD, *P*-value)					IC_50_μg/mL	SI
		12.5 μg/mL	25 μg/mL	50 μg/mL	100 μg/mL	200 μg/mL		
Leaf	ME	4.79 ± 0.38 0.0011	7.82 ± 2.12 0.012	10.03 ± 1.14 0.0028	17.72 ± 2.08 0.0027	23.38 ± 3.65 0.0054	>200	>8.33
	CH	0.00 ± 0.00 NS	0.00 ± 0.00 NS	0.00 ± 0.00 NS	4.12 ± 2.12 0.07 ^NS^	3.45 ± 2.32 0.2 ^NS^	ND	ND
	HE	4.77 ± 1.49 0.017	2.25 ± 0.36 0.0049	8.30 ± 0.83 0.0017	7.70 ± 0.57 0.0014	5.56 ± 0.69 0.017	>200	ND
	EA	0.00 ± 0.00 NS	0.00 ± 0.00 NS	10.36 ± 0.79 0.0010	20.38 ± 5.04 0.011	31.46 ± 0.97 0.0002	>200	>2.84
	AQ	0.00 ± 0.00 NS	4.01 ± 2.15 0.045	10.80 ± 2.53 0.0092	18.33 ± 0.98 0.0006	25.55 ± 1.50 0.0008	>200	>2.17
Bark	ME	0.00 ± 0.00 NS	4.71 ± 1.05 0.0087	13.05 ± 1.00 0.0010	19.64 ± 1.40 0.0010	29.61 ± 2.42 0.0014	>200	>17.13
	CH	0.00 ± 0.00 NS	0.00 ± 0.00 NS	4.25 ± 0.07 0.0000	7.74 ± 1.86 0.013	17.47 ± 2.08 0.0036	>200	00
	HE	0.00 ± 0.00 NS	2.25 ± 0.24 0.0023	4.69 ± 2.58 0.047	2.59 ± 0.93 0.066^NS^	5.06 ± 2.16 0.14 ^NS^	ND	ND
	EA	1.33 ± 0.22 0.0062	4.70 ± 0.84 0.0056	11.43 ± 2.75 0.0096	20.67 ± 2.21 0.0022	39.81 ± 3.33 0.0014	>200	>4.28
	AQ	0.00 ± 0.00 NS	0.00 ± 0.00 NS	0.00 ± 0.00 NS	1.30 ± 0.30 0.35 ^NS^	2.42 ± 1.02 0.84 ^NS^	ND	ND
Flower	ME	0.00 ± 0.00 NS	7.38 ± 2.22 0.015	15.36 ± 2.90 0.0060	22.31 ± 2.19 0.0018	34.58 ± 1.43 0.0004	>200	>6.25
	CH	0.00 ± 0.00 NS	0.00 ± 0.00 NS	0.00 ± 0.00 NS	1.30 ± 0.07 0.29 ^NS^	2.34 ± 1.10 0.85 ^NS^	ND	ND
	HE	2.62 ± 0.72 0.014	7.60 ± 1.46 0.0063	18.59 ± 0.78 0.0003	24.54 ± 3.77 0.0043	33.10 ± 2.82 0.0015	>200	00
	EA	0.00 ± 0.00 NS	0.00 ± 0.00 NS	0.00 ± 0.00 NS	0.00 ± 0.00 NS	1.60 ± 0.44 0.99 ^NS^	ND	ND
	AQ	8.25 ± 0.29 0.0002	0.00 ± 0.00 NS	7.58 ± 1.41 0.0059	5.56 ± 0.81 0.0063	6.54 ± 1.44 0.06 ^NS^	ND	ND
Root	ME	8.66 ± 1.93 0.0084	14.40 ± 1.22 0.0012	20.57 ± 0.86 0.0003	23.10 ± 3.64 0.0046	29.65 ± 2.88 0.0020	>200	7.79
	CH	0.00 ± 0.00 NS	2.18 ± 0.58 0.013	11.35 ± 2.47 0.0079	17.80 ± 2.10 0.0027	23.10 ± 2.06 0.0015	>200	ND
	HE	0.00 ± 0.00 NS	0.00 ± 0.00 NS	0.00 ± 0.00 NS	0.00 ± 0.00 NS	2.64 ± 0.49 0.92 ^NS^	ND	ND
	EA	4.28 ± 1.24 0.014	0.00 ± 0.00 NS	7.51 ± 2.14 0.014	3.42 ± 0.64 0.016	10.87 ± 0.89 0.0024	ND	ND
	AQ	0.00 ± 0.00 NS	0.00 ± 0.00 NS	12.56 ± 4.38 0.020	18.73 ± 2.06 0.0023	28.79 ± 3.43 0.0030	>200	>2.27
DMSO (Negative control)	–	0.40 ± 0.00	0.54 ± 0.11	0.60 ± 0.05	1.21 ± 0.42	1.56 ± 0.21	–	–
Ellipticine (Positive control)	–	–	–	–	–	–	0.59 ± 0.25	–

Values are represented as mean of 3 replicates ± standard deviation at 95% confidence interval with upper and lower limits and *P* - value is significant at <0.05 and <0.001, NS- not significant, ME- methanol, CH- chloroform, HE- hexane, EA- ethyl acetate, AQ- aqueous, SI- selective index (SI = IC_50_ THP-1 cell line/IC_50_ *P. f* 3D7 strain), ND- Not determinate, DMSO- Dimethyl sulphoxide

### Chemical injury to erythrocytes

The microscopic observation of uninfected erythrocytes incubated with the extracts of *Pongamia pinnata* and uninfected erythrocytes from the blank column of the 96-well plate showed no morphological differences after 48 h of incubation (Fig. 5). Hence, these extracts are not harmful to erythrocytes during the investigation and are safer to use as a remedy for malaria*.*

**Fig. 5:** Screening for chemical injury to erythrocytes after treatment of different crude extracts from *Pongamia pinnata* at higher concentration of 200 μg/mL (ME- methanol, CH- chloroform, HE- hexane, EA- ethyl acetate, AQ- aqueous)

### 4-Day suppressive test

The obtained results signify that, methanolic extracts of *Pongamia pinnata* displayed very good activity against *Plasmodium berghei* in vivo in BALB/c experimental mice. During the study period, the methanol extract of bark caused a moderately low (*P* < 0.05) and dose-dependent decrease in parasitemia unlike the chloroquine treated group, while the control negative group shown a daily increase in parasitemia.

During the early infection oral administration of 200, 400, 600, 800 and 1000 mg/kg body weight/day concentration of extract caused chemo-suppression of 14.59, 25.17, 36.71, 66.25 and 83.84% respectively on day-4 which was significant at *P* < 0.05 when compared to control negative. The standard drug chloroquine (5 mg/kg b.wt./day) caused 100% chemo-suppression which was highly significant when compared to the extract treated groups (Table 6). The highest concentration of extract (1000 mg/kg b.wt./day) shown 83.84% chemo-suppression which is almost like to that of standard drug chloroquine (5 mg/kg b.wt./day).

**Table 6:** Parasitemia, inhibition, survival time, body weight and packed cell volume in 4-day suppressive test after administration of methanolic bark extract of *Pongamia pinnata* against *Plasmodium berghei* infected BALB/c experimental mice

Test substance	Dose (mg/kg/day)	Parasitemia (%)	Inhibition (%)	Mean survival time (Days)	Weight on Day0 (g)	Weight on Day4 (g)	Change (%)	PCV on Day 0 (%)	PCV on Day 4 (%)	Reduction (%)
Methanol extract	200	38.29 ± 1.79 0.012*	14.59	10 ± 2.00 0.50^NS^	30.62 ± 1.22	30.13 ± 0.97 0.004*	1.63	42.16 ± 2.33	42.42 ± 1.15 0.018*	−0.49
	400	33.53 ± 0.43 0.0000*	25.17	13 ± 1.00 0.0011*	30.31 ± 2.33	31.08 ± 0.48 0.001*	3.23	42.42 ± 1.05	42.64 ± 0.28 0.013*	−0.43
	600	28.35 ± 1.81 0.0021*	36.71	17 ± 2.65 0.025*	30.51 ± 1.85	30.63 ± 0.79 0.003*	6.16	43.24 ± 1.65	44.02 ± 0.58 0.0022*	−1.46
	800	15.14 ± 1.06 0.0002*	66.25	22 ± 2.00 0.0057*	30.12 ± 1.48	30.72 ± 0.65 0.022*	−1.99	42.13 ± 2.03	43.36 ± 1.07 0.0084*	−2.35
	1000	07.24 ± 1.00 0.001*	83.84	26 ± 2.00 0.0032*	30.00 ± 3.21	31.35 ± 1.08 0.0004*	−4.53	43.63 ± 1.44	44.12 ± 2.59 0.037*	−0.91
Vehicle (−)	1 ml	44.81 ± 1.52	–	10 ± 1.00	30.23 ± 2.41	28.27 ± 2.56	6.48	43.00 ± 1.00	38.72 ± 1.87	8.07
Chloroquine (+)	5	0.00 ± 0.00	100	30 ± 0.00	30.24 ± 1.00	31.18 ± 1.23	−3.10	41.83 ± 2.46	44.21 ± 2.12	−4.59

The values are represented as mean of 3 values ± standard deviation and significant at *P < 0.05 (compared with negative control), NS- not significant, (−) Negative control, (+) Positive control

The comparative analysis indicated that, methanolic bark extract of *Pongamia pinnata* showed statistically significant difference on day-4 parasitemia at all dosages when compared to the negative control. The low level of parasitemia was observed at the highest dose (1000 mg/kg b.wt./day) of methanolic bark extract of *Pongamia pinnata* with 07.24% (Table 6) and statistically significant at *P* < 0.05.

The mean survival time (MST) of the chloroquine treated mice (control positive) was 30 days±0.00. The MST of infected mice (control negative) was ten days. The methanolic bark extract MST was significantly higher (*P* < 0.05) than the value of the negative control hence, the MST was lower than the standard drug chloroquine treated mice (Table 6).

In the 4-day suppressive test, all the doses of the extract showed a preventive effect on weight reduction and normalized the weight in infected mice at all dosages when compared to control negative group (Table 6). The methanolic bark extract exhibited protective activity against the reduction in packed cell volume (PCV) levels when compared to control negative (Table 6).

### Repository test

The methanol bark extract of *Pongamia pinnata* caused a moderately low (*P* < 0.05) and dose-dependent decrease in parasite counts unlike the chloroquine treated group, while the control group showed a daily increase in parasitemia. At 5 mg/kg b.wt./day, chloroquine produced 100% of chemosuppression (Table 7). The highest concentration of extract (1000 mg/kg b.wt./day) shown 87.47% chemo-suppression which was almost similar to that of standard drug chloroquine (5 mg/kg b.wt./day).

**Table 7:** Parasitemia, inhibition, survival time, body weight and packed cell volume in repository test after administration of methanolic bark extract of *Pongamia pinnata* against *Plasmodium berghei* infected BALB/c experimental mice

Test substance	Dose (mg/kg/day)	Parasitemia (%)	Inhibition (%)	Mean survival time (Days)	Weight on Day0 (g)	Weight on Day4 (g)	Change (%)	PCV on Day 0 (%)	PCV on Day 4 (%)	Reduction (%)
Methanol extract	200	52.27 ± 1.93 0.018*	10.57	10 ± 2.00 0.07^NS^	31.42 ± 1.53	30.75 ± 1.06 0.001*	2.13	45.21 ± 2.00	44.18 ± 1.90 0.04*	1.86
	400	44.62 ± 1.34 0.0008*	23.66	12 ± 1.34 0.04*	32.12 ± 0.85	32.53 ± 0.69 0.003*	−1.27	45.43. ± 1.65	45.12 ± 5.01 0.02*	0.55
	600	24.56 ± 3.69 0.0043*	57.98	15 ± 1.00 0.009*	30.31 ± 1.66	31.36 ± 0.79 0.004*	−3.46	44.82 ± 1.23	44.45 ± 0.73 0.03*	0.67
	800	15.94 ± 1.35 0.0000*	72.73	20 ± 2.55 0.0002*	31.09 ± 2.11	32.02 ± 0.84 0.002*	−2.99	46.05 ± 2.11	46.84 ± 1.12 0.003*	−1.40
	1000	7.32 ± 0.78 0.0000*	87.47	25 ± 0.00 0.0001*	32.00 ± 1.73	31.21 ± 1.63 0.001*	2.46	46.36 ± 0.56	45.73 ± 1.56 0.0083*	−0.79
Vehicle (−)	1 ml	58.45 ± 1.26	–	9 ± 1.85	31.63 ± 1.00	27.27 ± 0.89	13.78	44.72 ± 1.31	43.49 ± 1.82	2.25
Chloroquine (+)	5	00 ± 00	100	29 ± 1.38	31.43 ± 2.09	31.58 ± 1.32	−0.47	44.31 ± 1.06	46.45 ± 2.21	−3.94

The values are represented as mean of 3 values ± standard deviation and significant at *P < 0.05 (compared with negative control), NS- not significant, (−) Negative control, (+) Positive control

The comparative analysis indicated that, methanolic bark extract of *Pongamia pinnata* showed statistically significant difference in parasitemia compared to the negative control. The low level of parasitemia was observed at highest dose (1000 mg/kg b.wt./day) of methanolic bark extract of *Pongamia pinnata* with 7.32% (Table 7) and statistically significant at *P* < 0.05.

The mean survival time (MST) of the chloroquine treated mice (control positive) was 29 days. The MST of infected mice (control negative) was nine days. The MST of methanol bark extract treated mice was significantly higher (*P* < 0.05) than the value of the control negative mice which survived only for nine days hence the MST was lower than the standard drug chloroquine treated mice (Table 7).

During repository test, all the doses of the extract shown to have a preventive effect on weight reduction and normalized the weight in infected mice at all dose levels compared to negative control mice and the increase in body weight was not dose-dependent (Table 10). The methanolic bark extract exhibited protective activity against the reduction in PCV levels compared to control negative but it was not dose-dependent (Table 7).

### Curative test (Rane’s test)

Oral administration of 200, 400, 600, 800 and 1000 mg/kg b.wt./day concentration of methanolic bark extract of *Pongamia pinnata* suppressed parasitemia and was statistically significant at *P* < 0.05 when compared to negative control. The standard drug chloroquine (5 mg/kg b.wt./day) caused 100% chemo-suppression which was highly significant when compared to the extract treated groups (Table 12). The highest concentration of extract used (1000 mg/kg b.wt./day) showed 94.67% chemo-suppression which was almost like to that of standard drug chloroquine (5 mg/kg b.wt./day).

The comparative analysis indicated that, methanolic bark extract of *Pongamia pinnata* showed statistically significant difference in parasitemia at all dosages compared to the negative control. The low-level parasitemia was observed at the highest dose (1000 mg/kg b.wt./day) of methanolic bark extract of *Pongamia pinnata* with 2.12% (Table 8) and statistically significant at *P* < 0.05.

**Table 8:** Parasitemia, inhibition, survival time, body weight and packed cell volume in curative test after administration of methanolic bark extract of *Pongamia pinnata* against *Plasmodium berghei* infected BALB/c experimental mice

Test substance	Dose (mg/kg/day)	Parasitemia (%)	Inhibition (%)	Mean survival time (Days)	Weight on Day0 (g)	Weight on Day4 (g)	Change (%)	PCV on Day 0 (%)	PCV on Day 4 (%)	Reduction (%)
Methanol extract	200	23.45 ± 0.30 0.0014*	41.09	14.00 ± 2.00 0.06^NS^	29.21 ± 1.35	29.42 ± 1.11 0.004*	−0.71	39.42 ± 1.94	42.96 ± 2.87 0.007*	−8.98
	400	18.91 ± 1.18 0.0002*	52.49	18.00 ± 1.00 0.0004*	29.08 ± 2.34	29.53 ± 4.05 0.003*	−1.54	39.82 ± 2.11	43.40 ± 1.18 0.004*	−7.18
	600	11.28 ± 1.15 0.0001*	71.66	23.00 ± 2.00 0.0084*	28.30 ± 2.00	30.18 ± 1.98 0.005*	−6.64	38.19 ± 3.22	44.13 ± 3.98 0.001*	−12.32
	800	5.61 ± 0.48 0.0003*	85.90	27.00 ± 2.65 0.0081*	28.91 ± 1.23	29.26 ± 1.97 0.008*	−1.21	40.25 ± 1.58	42.44 ± 2.16 0.006*	−4.35
	1000	2.12 ± 0.03 0.0003*	94.67	29.00 ± 1.00 0.0000*	29.10 ± 2.11	31.47 ± 1.11 0.001*	−8.14	39.61 ± 1.33	44.18 ± 0.96 0.0008*	−8.43
Vehicle (−)	1 ml	39.81 ± 1.25	–	9.00 ± 1.58	29.31 ± 1.39	26.55 ± 1.56	9.41	38.32 ± 2.44	36.09 ± 1.88	5.87
Chloroquine (+)	5	00 ± 00	100	>30	30.22 ± 2.24	31.29 ± 2.11	−3.54	40.11 ± 3.21	43.54 ± 2.33	−6.84

The values are represented as mean of 3 values ± standard deviation and significant at *P < 0.05 (compared with negative control), NS- not significant, (−) Negative control, (+) Positive control

The MST of the chloroquine treated mice (control positive) was >30 days. The MST of infected mice (control negative) was nine days. The MST of methanolic bark extract treated mice was significantly higher (*P* < 0.05) than the control negative mice (Table 8).

During the established infection, all the doses of the extract showed a preventive effect on weight reduction and normalized the weight in infected mice at all dosages when compared to control negative group and the increase in body weight was not dose-dependent (Table 8). The methanolic bark extract exhibited protective activity against the reduction in PCV levels when compared to negative control but it was not dose-dependent (Table 8).

Thus, the inhibition of parasites during suppressive, repository and curative tests after treatment with the methanol bark extract of *Pongamia pinnata* against *Plasmodium berghei* at 1000 mg/kg b.wt./day is promising when compared with the control negative (Fig. 6). The comparative account of % of parasitemia, % of inhibition and mean survival time at 1000 mg/kg b.wt./day of the extract during 4-day suppressive, repository and curative tests is represented in Fig. 7.

**Fig. 6:** Microscopic observations after treatment with methanolic bark extract of *Pongamia pinnata* against *Plasmodium berghei* strain at the highest concentration (1000 mg/kg b.wt./day) with Giemsa(G) and Acridine Orange (AO) at 1000× magnification (R- ring stage, T- trophozoite, S- schizont, WBC- white blood cells)

**Fig. 7:** Graphical representation of % Parasitemia, % Inhibition and Mean Survival Time during 4-Day suppressive, Repository and Curative tests after administration of methanolic bark extract of *Pongamia pinnata* at 1000 mg/kg b.wt./day

The highest percentage of parasitemia levels were observed in control negative groups after inoculations of *P. berghei* parasites. Lowest parasitemia levels were observed in the group which was treated with chloroquine. Parasitemia in negative control mice was higher than all the treated groups. This had confirmed that all the treatments had an effect on the growth of *P. berghei* parasites in experimental mice. Parasitemia increased gradually in all the groups, and all the mice died on the10^th^ or 9th day in the negative control group. However, all the mice were alive and healthy up to day 30 in the positive control group.

Finally it is established that, the methanolic bark extract of *Pongamia pinnata* (Pierre) at 1000 mg/kg b.wt./day has shown highest percent of inhibition, low parasitemia level and more survival time in experimental BALB/c mice.

## Discussion

The present investigation had revealed that, methanol bark extract of *Pongamia pinnata* (IC_50 =_ 11.67 μg/mL) had shown maximum antiplasmodial and synergistic activity of one or more phytochemical constituents amongst all the tested extracts according to the classification of Rasoanaivo et al. [19]. The results of our study are in consistent with the outcomes of peer researchers who reported the antiplasmodial activity of several plants including polyherbal extracts [24, 31–36].

Our results are closely related to the previous reports of Simosen et al. [18] who reported the antimalarial activity of *Pongamia pinnata* ethanol extracts in different plant parts such as leaves, bark and seeds. Among these extracts, bark and leaf shows good antiplasmodial activity with the IC_50_ values of 25 μg/mL and 24 μg/mL respectively; remaining seed extracts showed mild activity with the IC_50_ value of 79 μg/mL. Recently Singh et al. [37] reported antimalarial activity of *Pongamia pinnata* ethanol extracts of leaves and bark along with 22 native medicinal plants from Chhotanagapur Plateau, Jharkhand, India against CQ-sensitive *P. f.* 3D7 and CQ-resistant *P. f.* INDO strains. The IC_50_ values of leaves and bark have shown good antiplasmodial activity with 22.8 μg/mL and 9.5 μg/mL respectively.

Guna et al. [1] reported the larvicidal activity of *Pongamia pinnata* methanol and hydroalcoholic extracts against three mosquito vectors *Culex quinquefasciatus*, *Aedes aegypti* and *Anopheles stephensi*. In their studies, the hydroalcoholic extract of *Pongamia pinnata* showed a significant mortality in three mosquito larvae. The above reports strongly support the present plant *Pongamia pinnata* showing promising growth inhibition of *Plasmodium falciparum.* In contrast to this, Mbatchi et al. [38] studied the antimalarial activity of *Millettia versicolor;* Millettia is a synonym of Pongamia whose plant extracts were inactive showing the IC_50_ > 100.

Bagavan et al. [14] have also conducted similar work and reported the antimalarial activity of *Citrus sinensis* (peel), *Leucas aspera, Ocimum sanctum, Phyllanthus acidus* (leaf), and *Terminalia chebula* (seed) in different extracts such as hexane, chloroform, ethyl acetate, acetone, and methanol against chloroquine-sensitive (3D7) strain of *P. falciparum* and studied cytotoxicity on HEp-2 and Vero cell lines. Out of the 25 extracts tested, the ethyl acetate and methanol extracts of leaf of *L. aspera*; ethyl acetate, acetone and methanol extracts of leaf of *P. acidus*; and acetone extract of seed of *T. chebula* has good antiplasmodial activity (IC_50_7.81, 22.76, 9.37, 14.65, 12.68 and 4.76 μg/mL) with selectivity indices 5.43, 2.04, 4.88, 3.35, 3.42, and 9.97 for HEp-2 and >5.79, >2.20, >11.75, >3.41, >3.94, and >7.38 for Vero cells respectively. These analyses have revealed for the first time that the components present in the solvent extracts of *L. aspera*, *P. acidus* and *T. chebula* have antiplasmodial activity.

Chenniappan and Kadarai [39] tested the antimalarial activity of 50 traditionally used Western Ghats plants alone and in combination with chloroquine against CQ-resistant *Plasmodium falciparum* strains from India. Out of 200 extracts, 29 extracts showed significantly high in vitro antiplasmodial activity with IC_50_ values ranging from 3.96 to 4.85 μg/mL, 53 extracts demonstrated significantly good in vitro antiplasmodial activity with IC_50_ values ranging from 5.02 to 9.87 μg/mL and 28 extracts shown significantly moderate in vitro antiplasmodial activity with IC_50_ values ranging from 10.87 to 14 μg/mL respectively. Our results are closely related to their results. In combination with CQ, 103 extracts showed significant synergistic in vitro antiplasmodial activities with synergistic factor values ranging from 1.03 to 1.92 and these activities were up to a fold higher with CQ, suggesting synergistic interaction of the chloroquine and the plant extract.

Kirira et al. [40] evaluated the activity of the aqueous, chloroform and methanol extracts from *Zanthoxylum usambarense* on *P*. *falciparum* showed the IC_50_ values of 6.04, 3.14 and 6.12 μg/ml respectively and the IC_50_ value for the aqueous extract from the same plant fell between 6 and 15 μg/mL against both CQ-sensitive and resistant *P*. *falciparum* strains, while that of methanolic extract was found to be lower than 6 μg/mL and these results coincide with our results.

The in vitro antiplasmodial activity the plant extracts of *Pongamia pinnata* may be because of the presence of strong phytochemical constituents such as phenols, flavonoids, coumarins and alkaloids. Since, alkaloids are the major classes of compounds possessing antimalarial activity; quinine is one of the important and oldest antimalarial drugs which belong to this class of compounds [41]. Apart from alkaloids, the presence of most important compounds such as coumarins, phenols, carbohydrates, terpenoids and flavonoids in the plant extracts under the study said to possess strong antiplasmodial activities. This is supported by the findings that alkaloids, flavonoids and sesquitepenes are the potent secondary metabolites of plant with broad spectrum of bioactive functions [42].

Biological activity is recognized as the presence of various secondary metabolites in plants [41]. In view of this, it is visualized that any one of the classes of compounds may be responsible for the activity. Cytotoxicity is also attributed to the occurrence of diverse secondary metabolites found in plant extracts. Not only their presence, but also the quantity of the phytochemical constituents in a given plant extract will determine the extent of its bioactivity. Also, the occurrence of more than one class of secondary metabolites in a particular plant extract determines the nature and magnitude of its biological activity [43]. Hence, various chemical compounds may be present in high concentration in methanol bark extract of *Pongamia pinnata* which may be responsible for their high antimalarial activity. The polysaccharides of higher plants possessed immunostimulatory, anticomplementary, antiinflammatory, hypoglycemic and antiviral activities [35].

BSLA indicates general toxicity and can be used for the detection of antitumor and pesticidal compounds. The low cost and ease of performing the assay and the commercial availability of inexpensive brine shrimp eggs makes BSLA a very useful bench top method. In vivo and in vitro cytotoxicity test has been successfully used as a preliminary study for cytotoxic and antitumor agents. Thus, the findings of this present study provides baseline information on the majority of promising plant species that could be of used as a basis for the development of new tools of a considerable therapeutic importance [44].

The general toxicity activity was considered non-toxic when the LC_50_ is greater than 1000, weak when the LC_50_ is from 500 to 1000 μg/mL, moderate when LC_50_ is from100 to 500 μg/mL and strong when the LC_50_ is below 100 μg/mL [45]. In the present observation, the plant extracts of methanol, ethyl acetate and aqueous have shown good antiplasmodial activity also shown LC_50_ values ranging from 500 to 1475 μg/mL. According to the above categorization, these have weaker toxic properties hence these are safer for therapies. Non-toxicity of the tested plant extracts suggest that the plants have a potential to inhibit the growth of Plasmodium parasites which is not associated with their inherent toxicity. In contrast to this, high cytotoxicity of Kenyan medicinal plants on brine shrimp larvae was reported by Nguta et al. [46].

The cytotoxic effect in vitro against THP-1 cell lines revealed that out of 20 extracts, all extracts showed IC_50_ > 200 μg/mL. The cytotoxicity of more than 20 μg/mL is considered as non-toxic to animals which are safer for further studies. Based on the above, all the plant extracts are not harmful and safer for further research and therapeutic studies. The SI of most of the extracts showed >10 for both BSLA and THP-1 cell line cytotoxicity studies. The SI is defined as the ratio of the cytotoxicity on the brine shrimp to the antiplasmodial activity. Those that showed high SI (>10) should offer the potential for safer therapy [47].

Also, none of the test extracts of three experimental plants have shown any of the chemical injuries to the erythrocytic membrane throughout the experimentation. The erythrocytic membrane is a fragile structure that can be significantly changed by drug interactions. The mechanical permanence of the erythrocytic membrane is an excellent indicator of in vitro studies for cytotoxicity screening because of its structural dynamics favoring interactions with drugs and this signifies that, the possible use of these extracts as an antiplasmodial drug in future. The mechanism of action might be due to the inhibition of hemozoin biocrystallization by the alkaloids and inhibition of protein synthesis by triterpenoids [48].

The in vivo model was engaged for this study for the reason that it takes into account the possible pro-drug effect and the possible involvement of the immune system in the eradication of infection. *P. berghei* ANKA was used in the prediction of treatment outcomes and for this reason it was an appropriate parasite for the study. Additionally, several conventional antimalarial agents such as chloroquine, halofantrine, mefloquine and more recently artemisinin derivatives have been identified using a rodent model of malaria [49]. The 4-day suppressive test, which mainly evaluates the antimalarial activity of extracts on early infections, Rane’s test, which evaluates the curative capability of extracts on established infections, and repository test which studies the prophylatic activity of extracts are the common tests for antimalarial drug screening used in the present study. In the three methods, the most reliable parameter is a determination of percent inhibition of parasitemia. A mean parasitemia level ≥ 90% to that of mock-treated control animals usually indicates that the test compound is active in standard screening studies [45].

Anemia, loss of body weight and body temperature reduction are the common symptoms of malaria infected mice [45]. Thus ideal antimalarial agents obtained from plants are expected to prevent body weight loss in infected mice due to the rise in parasitemia. Despite the fact that the increase in weight was not consistent with an increase in dose, the crude extract of *Pongamia pinnata* significantly prevented weight loss associated with the decrease in parasitemia level in suppressive, repository and curative tests to *P. berghei*. The preventive effect of extract might be due to the presence of saponins, flavonoids, glycosides and phenolic compounds found in the crude extract [50].

PCV was measured to evaluate the efficacy of the methanol extract in preventing hemolysis due to escalating parasitemia level. The fundamental cause of anemia incorporates the following mechanisms: the clearance and or destruction of infected RBCs, the clearance of uninfected RBCs, erythropoietic suppression and dyserythropoiesis. Each of these mechanisms has been concerned with both human and mouse malarial anemia [30]. According to the present study methanol extract did not show any preventive effect on PCV reduction in suppressive, repository and curative tests. However, the reduction of PCV is a slight variant when compared to the controls.

In vivo antiplasmodial activity can be classified as moderate, good and very good if an extract demonstrated the percentage of parasitemia suppression equal to or greater than 50% at a dose of 500, 250 and 100 mg/kg b.wt./day respectively [45]. Based on this classification, the crude extract of the studied plant, *Pongamia pinnata* has shown good antiplasmodial activity.

Drugs lead to decreased parasitemia and subsequent recovery of symptomatic malaria. They also reduce parasitemia through different ways like reducing parasite nutrient intake, interfering with parasite metabolic pathways like a heame metabolic pathway which is involved in the metabolism of iron [51]. Drugs also negatively influence the parasite reproduction and growth [30]. The plant extract reduced the level of parasitemia and increased the mice survival time. Chloroquine had a good chemo-suppression of 100% as determined by post-infection and a 100% survival rate on post-infection.

Moreover, our present observation is also supported by Chand et al. [26] who reported that the ethanolic extract of the leaves of *Ajuga bracteosa* has shown to reduce the number of Plasmodium parasites in a mouse model. Previous studies have shown that water and methanolic stem bark extracts of *Zanthoxylum chalybeum* have significant in vitro antiplasmodial activity against CQ-sensitive and CQ-resistance strains of *P. falciparum* [52], which corroborates with the findings of the present study that the methanolic bark extract of *Pongamia pinnata* has exhibited significant in vitro antimalarial activity.

Previously, Ogbuehi et al. [53] reported the suppressive, repository and therapeutic activity of the methanolic root extracts of *Anthocleista noblis, Nauclea latifolia* and *Napoleona imperialis* from south-east medicinal plants in Nigeria promisingly reduced the parasitemia. Anosa et al. [54] studied in vivo antiplasmodial activity of ethanolic extract of stem bark of *Enantia polycarpa* in mice infected with *Plasmodium berghei*. The extracts exhibited promising activity against both the early and established infection and achieved 75.8% and 72% chemo-suppression and increased the MST after administration. Thus, the previous reports on in vivo antimalarial activity strongly support and corroborates with the present findings that the methanolic bark extract of *Pongamia pinnata* has exhibited promising in vivo antimalarial activity in *P. berghei* infected BALB/c experimental mice.

## Conclusions

The present investigation revealed that, out of 20 extracts of the studied plant, *Pongamia pinnata* the methanolic bark extract exhibited the most potent antimalarial activity against *Plasmodium falciparum* in vitro and against *Plasmodium berghei* in vivo*.* Moreover, these plant extracts does not exhibited toxicity both under in vivo and in vitro conditions against brine shrimp larvae and THP-1 cell line respectively. Thus, the present work is giving the scope of using these compounds or substances for further therapeutic studies for new drug formulations. Hence, more research is needed to identify and characterize the potent molecules that suppress the malaria parasite for new drug therapies in view of growing resistance to malaria.

## Abbreviations

AIDS: Acquired immune deficiency syndrome
AQ: Aqueous
BSLA: Brine shrimp lethality assay
CH: Chloroform
CNS: Central nervous system
CPM: Counts per minute
CQ: Chloroquine
DMSO: Dimethyl sulfoxide
EA: Ethyl acetate
h: Hours
HE: Hexane
IC: Inhibitory concentrations
LC: Lethal concentration
ME: Methanol
ND: Not determinate
*P. falciparum*: *Plasmodium falciparum*
PBS: Phosphate buffered saline
PCV: Packed cell volume
RBC: Red blood cells
RPMI medium: Roswell park memorial institute medium
UV: Ultra violet
WHO: World health organization
